# Systematic Review of the Efficacy and Safety of Traditional Chinese Medicine Granules Associated with Hormone When Treating Primary Nephrotic Syndrome in Children

**DOI:** 10.1155/2022/2520367

**Published:** 2022-09-27

**Authors:** Li Zhang, Lei Chen

**Affiliations:** ^1^Department of Pediatrics, Qilu Medical University, Zibo, Shandong, China; ^2^Department of Surgery, Qilu Medical University, Zibo, Shandong, China

## Abstract

**Objective:**

To systematically evaluate the efficacy and safety of traditional Chinese medicine (TCM) granules associated with hormones when treating primary nephrotic syndrome (PNS) in children.

**Methods:**

Search online databases such as PubMed, EMBASE, ScienceDirect, Cochrane Library, China Knowledge Network Database (CNKI), China VIP Database, Wanfang Database, and China Biomedical Literature Database (CBM) to search for information on the use of hormone-related Chinese medicine granules in the treatment of children with PNS controlled trials. Retrieval time was limited to the period from the date the database was established to the present. Separately, two researchers gathered the data. Statistical software RevMan5.4 was adopted to estimate bias risk in accordance with the Cochrane Handbook 5.3 standard.

**Results:**

Finally, 7 articles were selected with a total sample size of 487 cases. The infection rate, recurrence rate, and adverse reaction rate after treatment were analyzed by meta-analysis. The infection rate and recurrence rate in the study group were notably lower, and the difference was statistically significant (*P* < 0.05). However, the incidence of adverse reactions exhibited not notably different (*P* > 0.05). The levels of albumin and blood cholesterol after treatment indicated no statistical difference between the levels (*P* > 0.05). Meta-analysis was performed on the time to negative urine protein and the time to edema subsidence after treatment. The urine protein negative time and edema subsidence time of the study group were shorter after treatment, but the difference exhibited not notable (*P* > 0.05). Meta-analysis was performed on the dosage of glucocorticoids after treatment. The dosage of glucocorticoid in the study group was notably lower, and the difference was statistically significant (*P* < 0.05). The levels of T lymphocytes after treatment were analyzed by meta. T lymphoid level in the study group was notably better after treatment, and the difference was statistically significant (*P* < 0.05). Further subgroup analysis indicated that the levels of CD3+ and CD4+ in the study group were higher after treatment (*P* < 0.05), and there exhibited no statistical difference in the levels of CD8+, CD4/CD8+, and CD19 (*P* > 0.05). Immunoglobulin levels in the study group after treatment were notably better, and the difference was statistically significant (*P* < 0.05). Further subgroup analysis indicated that the levels of IgA, IgM, and IgG in the study group were notably higher after treatment, and the difference was statistically significant (*P* < 0.05).

**Conclusion:**

Huai Qi Huang can reduce the recurrence rate of PNS children and the incidence of infection and the dosage of prednisone. A long-term application can improve the cellular and humoral immune function of children with PNS. It has high treatment safety and has no notable effect on plasma cholesterol levels, so it is suitable for clinical application.

## 1. Introduction

The increased permeability of the glomerular filtration membrane to plasma proteins and the loss of a large amount of plasma proteins from the urine cause nephrotic syndrome (NS). NS is a clinical syndrome characterized by a series of pathophysiological changes. Proteinuria, hypoalbuminemia, hyperlipidemia, and edema are common symptoms in children suffering from a glomerular disease. In pediatric kidney disease, the incidence of NS is second only to acute nephritis [1]. NS can be assigned into three types, including congenital, primary, and secondary, among which primary nephrotic syndrome (PNS) is the most common, accounting for about 90% of all children's NS [2]. According to US statistics, the annual incidence of PNS in children is (2–4)/100,000, and the prevalence is 16/100,000 [3, 4]. Recent statistics have reported that PNS can account for about 20.0% of the total number of hospitalized children with urinary tract diseases in the same period [5]. The advantages of TCM when treating PNS in children are gradually revealed. TCM treatment follows the method of syndrome differentiation and treatment. It has attached importance to improving children's clinical symptoms and signs and reducing adverse reactions of hormones.

Children with cellular and humoral immune disorders are at an increased risk for developing PNS, according to related studies [6]. Another literature reported that hypo-immunoglobulin G (Immunoglobulin G, IgG) hyperemia is a high-risk factor for NS. And hypoIgG hyperemia in NS is also a cause of secondary infection and recurrent episodes of PNS [7]. Clinically, glucocorticoid is the first choice to treat PNS. Although it has a certain therapeutic effect, the patients treated with corticosteroids alone have a higher recurrence rate and greater side effects, resulting in hormone dependence. Some children have repeated illnesses and protracted disease courses, which seriously affect their health.

Rhizoma Polygonatum has the function of tonifying the kidney. Chinese wolfberry is an obviously adopted TCM for tonifying the liver and kidney. Previous studies have testified that it includes beet thrift, polysaccharide, crude fat, crude protein, carotene, vitamin A, C, B1, B2, and other nutrients. Huai Qi Huang granule is a granule made of Huaier fungus associated with Chinese wolfberry and Polygonatum. The main component of Sophora fungus is a new fungal drug produced by solid fermentation engineering from Fructus Sophorae mycelium. Its main component, Sophora fungus polysaccharide (PS2T), is a protein composed of 6 kinds of monosaccharides associated with 18 kinds of amino acids and contains mineral elements. Polysaccharides have immune activity and can improve the nonspecific anti-infection ability of the body. PS2T is a highly active biological response regulator, which can stimulate many links in the body's immune system, thus improving the body's immunity [8, 9]. Huai Qi Huang granule can notably improve the immune function of PNS patients, but the efficacy and safety of TCM when treating PNS patients have not been internationally recognized, which needs to be supported by high-quality research evidence. It can improve hematopoiesis, antiaging, antimutation, antitumor, antifatty liver, and hypoglycemic effects. Chinese wolfberry is often used to treat yin deficiency in the liver and kidney, sore waist and knees, dizziness, forgetfulness, dizziness, tears, thirst, spermatorrhea, and other diseases. It has been reported that Huai Qi Huang granule can reduce the incidence of infection and recurrence in patients with NS [10, 11]. It has also been reported that the Huai Qi Huang granule can reduce the excretion of urinary protein [12]. In addition, there are great differences between different research designs and a variety of evaluation indicators, with the effectiveness of literature or the improvement of an evaluation index to explain the clinical efficacy of TCM granule treatment. The results are not convincing, and many research results are not consistent. Therefore, this study made a systematic, quantitative and comprehensive analysis of the results of similar independent studies through meta-analysis. This study was to systematically evaluate the efficacy and safety of traditional Chinese medicine (TCM) granules associated with hormones when treating primary nephrotic syndrome (PNS) in children.

## 2. Research Contents and Methods

### 2.1. The Sources and Retrieval Methods of Documents

Search online databases such as PubMed, EMBASE, ScienceDirect, Cochrane Library, China Knowledge Network Database (CNKI), China VIP Database, Wanfang Database, and China Biomedical Literature Database (CBM) to search for information on the use of hormone-related Chinese medicine granules in the treatment of children with PNS controlled trials. And relevant data about the use of TCM granules associated with hormones to treat PNS in children were harvested. A literature search was carried out when forming free words and subject words, with the keywords of TCM granules, hormone therapy, PNS in children, efficacy, safety, TCM granules, hormone therapy, and PNS in children from January 2010 to March 2022.

### 2.2. Literature Inclusion and Exclusion Criteria

#### 2.2.1. Literature Inclusion Criteria

Inclusion criteria were as follows: (1) research types: all the controlled trials (CT) of Chinese herbal granules associated with hormones when treating PNS in children. The languages were Chinese and English; (2) subjects: children with PNS, the diagnostic criteria referred to the “evidence-based guidelines for diagnosis and treatment of Common Renal Diseases in Children (trial)” formulated by the Chinese Medical Pediatrics Association [13]; (3) intervention: the study group received TCM granules associated with hormone treatment, while the control group only received hormone treatment. Indications of TCM granule associated with hormones when treating PNS in children: the children were not allergic to experimental drugs, were not complicated with other severe somatic or mental diseases and were not treated with other drugs at the same time.

### 2.3. Literature Exclusion Standard

Exclusion criteria were as follows: (1) the data report was incomplete and the data could not be used; (2) the repeated research content was taken from the latest research; (3) the evaluation of the curative effect of the study was not notable.

### 2.4. Quality Evaluation and Data Extraction

1. Bias risk assessment contained in the study: for the evaluation, a bias risk assessment tool recommended by Cochrane System Review Manual 5.3 was adopted.
2. Literature screening and data extraction: independently, two researchers screened literature, gathered data, assessed quality, and cross-checked results. Note Express document management software and Excel office software were used to manage and extract research data. If the data contained in the literature was incomplete, the author of this article would be contacted to supplement it. The content of data extraction contained (1) basic information: author, publication time, number of cases; (2) intervention: plan, course of treatment; (3) outcome index.

### 2.5. Statistical Processing

The standardized mean difference (SMD) with Hedges' g was chosen as the measure of the effect. The effect size was calculated using a random-effects model with a restricted maximum-likelihood (REML) and considered a large, moderate, and small effect with respect to the SMD values of 0.8, 0.5, and 0.2, respectively. The heterogeneity among the studies included in a meta-analysis was assessed using Cochrane's Q, tau-squared, and I-squared (I2). Cochrane's Q test quantifies total variance and generates a *P*-value that determines the heterogeneity is present. Tau-squared indicates the true variance which is the between-study variance, while I2 represents the percentage of the total variance that is due to the true variance. The degree of heterogeneity is said to be low, moderate, and high, with I2 values of 25%, 50%, and 75%. RevMan 5.3 software was adopted for meta-analysis. HR and its 95% CI were employed as effect analysis statistics for OS and PFS, and risk ratio and 95% CI were employed as effect analysis statistics for binary variables. *P* and *I*^2^ values in heterogeneity test results were adopted to determine whether there was statistical heterogeneity among the results. *P* > 0.10, *I*^2^ < 50% indicated that there was no statistical heterogeneity among the research results, and a fixed effect model was used for combined analysis. *P* ≤ 0.10, *I*^2^ ≥ 50% indicated statistical heterogeneity among the research results, and a random-effects model was adopted for combined analysis. The test level of the meta-analysis was set as *α* = 0.05. Eggers' test was used to examine the funnel plot asymmetry. Whenever this test was significant with a *P* value of less than 0.1, we used the trim and fill method to correct the funnel plot and adjust the effect size for potential publication bias.

## 3. Results and Analysis

### 3.1. The Results of Literature Retrieval and the Basic Situation of Literature Inclusion

We used a computer database to retrieve 1832 articles, 441 articles were eliminated after removing repeated studies and 134 were retrieved by reading the titles and abstracts, after excluding irrelevant studies, reviews, case reports, and noncontrol literature, 98 articles were initially contained, and finally contained 7 articles [14–20]. The meta-analysis covered 487 samples in total. All results were shown in Figure 1 and Table 1.

### 3.2. Evaluation of the Quality of the Methodology Contained in the Literature

The seven CT articles included in this meta-analysis reported the baseline health status of the patients. Three articles did not specify the randomized method, although all other articles provided detailed intervention measures. According to the Jadad scale, it can be seen that 7 articles all scored ≤ 2 points. All results were shown in Figures 2 and 3.

### 3.3. Meta-Analysis Result

#### 3.3.1. Infection Rate

There were 7 studies contained in this study with 487 samples. Meta-analysis was performed on the infection rate. The results of the heterogeneity test indicated that (Figure 4) Chi^2^ = 1.63, df = 3, *P* = 0.65, and *I*^2^ = 0%, indicating that the research data contained in the study showed distinct heterogeneity. Using the fixed effect model analysis, it could be noticed that the infection rate of the research group after treatment was notably lower, and the difference was statistically significant (*P* < 0.05). All results were shown in Figure 4.

#### 3.3.2. Relapse Rate

A meta-analysis was performed on the recurrence rate after treatment. The results of the heterogeneity test indicated that (Figure 5) Chi^2^ = 4.10, df = 3, *P* = 0.25, and *I*^2^ = 27%, indicating that the research data contained in the study showed distinct heterogeneity. The fixed effect model analysis shows that the recurrence rate of the research group was notably lower, and the difference was statistically significant (*P* < 0.05). All results were shown in Figure 5.

#### 3.3.3. Incidence of Adverse Reactions

A meta-analysis was performed on the incidence of adverse reactions after treatment. The results of the heterogeneity test indicated that (Figure 6) Chi^2^ = 0.98, df = 1, *P* = 0.32, and *I*^2^ = 0%, indicating that the research data contained in the study showed distinct heterogeneity. No notable difference was found in the incidence of adverse reactions after treatment (*P* > 0.05). All results were shown in Figure 6.

#### 3.3.4. Serum Albumin

The meta-analysis of serum albumin levels after treatment was carried out. The results of the heterogeneity test indicated that (Figure 7) Chi^2^ = 41.22, df = 3, *P* < 0.00001, and *I*^2^ = 93%, indicating that the research data contained in the study showed distinct heterogeneity. The albumin level of the research group after treatment was higher, with no statistically notable (*P* > 0.05). All results were shown in Figure 7.

#### 3.3.5. Blood Cholesterol

Meta-analysis was performed on the blood cholesterol levels after treatment. The results of the heterogeneity test indicated that (Figure 8) Chi^2^ = 3.70, df = 2, *P* = 0.16, *I*^2^ = 46%. No notable difference in blood cholesterol levels after treatment (*P* > 0.05). All results were shown in Figure 8.

#### 3.3.6. Urinary Protein Negative Time

A meta-analysis was performed on the time of urine protein conversion to negative after treatment. The results of the heterogeneity test indicated that (Figure 9) Chi^2^ = 201.83, df = 3, *P* < 0.00001, and *I*^2^ = 99%. The urine protein negative time in the study group after treatment was shorter (*P* > 0.05). All results were shown in Figure 9.

#### 3.3.7. Edema Regression Time

A meta-analysis was performed on the edema subsidence time after treatment. The results of the heterogeneity test indicated that (Figure 10) Chi^2^ = 65.90, df = 2, *P* < 0.00001, and *I*^2^ = 97%. The random effect model analysis indicated that the edema subsidence time in the study group was shorter after treatment (*P* > 0.05). All results were shown in Figure 10.

#### 3.3.8. Glucocorticoid Dosage

A meta-analysis was performed on the dosage of glucocorticoids. The results of the heterogeneity test indicated that Chi^2^ = 0.45, df = 2, *P* = 0.80 > 0.05, and *I*^2^ = 0%. The dosage of glucocorticoid in the study group was notably lower, and the difference was statistically significant (*P* < 0.05). All results were shown in Figure 11.

#### 3.3.9. T Lymphocyte Level

A meta-analysis was performed on the levels of T lymphocytes after treatment. The results of the heterogeneity test indicated that (Figure 12) Chi^2^ = 586.77, df = 21, *P* < 0.00001, and *I*^2^ = 96%. T lymphocyte level in the study group after treatment was notably better, and the difference was statistically significant (*P* < 0.05). Further subgroup analysis indicated that the levels of CD3+ and CD4+ in the study group were higher after treatment, and the difference was statistically significant (*P* < 0.05). No notable difference was discovered in the levels of CD8+, CD4/CD8+, and CD19 (*P* > 0.05). All results were shown in Figure 12.

#### 3.3.10. Immunoglobulin Level

From the heterogeneity test results can be seen (Figure 13) Chi^2^ = 232.64, df = 14, *P* < 0.00001, *I*^2^ = 94%, indicating that the research data contained in the study showed distinct heterogeneity. Random effect model analysis indicated that the improvement effect of immunoglobulin levels in the study group was notably better after treatment, and the difference was statistically significant (*P* < 0.05). Further subgroup analysis indicated that the levels of IgA, IgM, and IgG in the study group were notably higher after treatment, and the difference was statistically significant (*P* < 0.05). All results were shown in Figure 13.

#### 3.3.11. Publication Bias Analysis

Publication bias analysis was conducted on the studies contained in each outcome index. The results indicated that except for the recurrence rate, the possibility of publication bias was small. The funnel chart affecting the recurrence rate was basically symmetrical, but the results of Egger's test and Begg's test indicated that there exhibited publication bias. There exhibited no notable change in the effect before and after trimming, indicating that the meta result was robust. All results were shown in Figure 14.

## 4. Analysis and Discussion

This study was to systematically evaluate the efficacy and safety of traditional Chinese medicine (TCM) granules associated with hormones when treating primary nephrotic syndrome (PNS) in children. At present, its pathogenesis and cause are not fully understood. Related studies have confirmed that in children with NS, CD3 and CD4 decreased notably and CD8 increased notably after the disease entered the active stage, while the aforementioned indexes changed on the contrary in the remission stage [21]. This result has confirmed that there is a cellular dysfunction in children with NS with an abnormal distribution of T cell subsets. Other scholars found that among the changes in humoral immune indexes in children with NS. One of the most obvious and serious signs is the serious decrease of IgG. After the disease entered the active stage, IgG decreased notably with the gradual improvement of the condition [22]. During the acute attack of children with NS, the loss of immunoglobulin in urine is more serious. The function of cellular and humoral immunity is more disordered, and the risk of infection is notably increased. At present, glucocorticoid is still the first choice to treat NS. Long-term use of corticosteroids will inhibit abnormal immunity, damage normal immune function, reduce body defense and increase the risk of infection. PNS is one of the obvious renal diseases in children. In this clinical syndrome, the permeability of the glomerular filtration membrane increases, resulting in a loss of plasma protein in the urine. The notable characteristics of the disease are hypoproteinemia, massive proteinuria, hyperlipidemia, and a certain degree of edema. The infection will lead to recurrent attacks and increase the mortality of children. Therefore, hormone therapy should be associated with immunomodulator therapy to regulate immunity and reduce the recurrence rate of infection and nephropathy.

The production of *α* and *γ*-INF is induced, cooperating with NK cells, which can directly inhibit tumor growth, accelerate tumor cell apoptosis and necrosis, improve cellular and humoral immune function, and thus regulate the imbalance of immune cells [23]. The active ingredient of Lycium barbarum is Lycium barbarum polysaccharide. Its modern pharmacological effect is to scavenge excess free radicals to delay aging, protect islet cell function, reduce blood sugar, promote immune cell activity, enhance phagocyte, and complement activity to improve immunity [24]. Huai Qi Huang granule is composed of Sophora fungus, Chinese wolfberry, and Polygonatum. *Sophora frutescens* is a kind of fungus, which mainly grows on the trunk of *Sophora japonica*, *Robinia pseudoacacia*, and sandalwood. Its main chemical composition is Sophora polysaccharide protein, which is composed of 6 kinds of monosaccharides and 18 kinds of amino acids. It is a highly active biological response regulator, which can stimulate many links in the body's immune system, increase the proliferation of T cells and strengthen the phagocytic function of macrophages. The main pharmacological effects of Polygonatum are regulating immunity, improving memory, anticancer, antiaging, reducing blood sugar, anti-inflammation, prevention and treatment of infection, and so on [25, 26]. From the literature contained in this study, a large number of studies on Huai Qi Huang granule associated with hormone when treating PNS patients have been carried out in China, including randomized controlled, double-blind, and multicenter high-level studies, which can show that Huai Qi Huang granule associated with hormone has high clinical value when treating PNS patients.

This study finally contained 7 articles with a total of 487 samples. The infection in the research group after treatment, rate, and recurrence rate were notably lower (*P* < 0.05), but the incidence of adverse reactions was not notably different (*P* > 0.05). This indicated that Huai Qi Huang granule associated with hormone treatment could notably reduce the infection rate and recurrence rate of PNS patients, which would not notably increase adverse reactions. Children with PNS are very susceptible to various infections. Though the infection is not severe, it often induces the recurrence of PNS or affects its efficacy. It is confirmed that Huai Qi Huang granule associated with hormone treatment has a good anti-inflammatory effect, which can effectively avoid the occurrence of infection, but also can play a good long-term effect. Moreover, the safety of the combination of the two drugs was higher, and the risk of adverse reactions in children was lower, which was suitable for young people. The main reason for the higher safety is that the age factor of the children has been taken into account when choosing hormones. The safe hormone can be selected for treatment, while Huai Qi Huang granule belongs to proprietary Chinese medicine preparation.

In this study, the levels of albumin and blood cholesterol after treatment were not statistically different. It is suggested that Huai Qi Huang granule has no effect on albumin and plasma cholesterol levels in children with PNS, which is consistent with previous studies. The research of Sun Wen in Pediatrics Hospital of Fudan University suggested that Huai Qi Huang granule could maintain the integrity of podocyte diaphragm by upregulating the expression of nephrin and podocin on the hiatus diaphragm, reduce the damage of glomerular filtration barrier, and increase serum albumin [27]. Huai Qi Huang granule is a kind of Chinese patent medicine with high safety. From the analysis of drug composition, it can be known that it will not have a great impact on blood indexes such as albumin and cholesterol, which has been confirmed by many clinical studies in the past.

The application of Huai Qi Huang granule can also reduce the amount of hormone used in the maintenance period, mainly because it can play a synergistic effect in combination with hormones, maximize clinical efficacy, and improve the condition of children faster and better. As a result, the amount of hormones will be greatly reduced. CD3+, CD4+, and CD8+ are indexes reflecting the cellular immune function of the body, and IgG is a vital index reflecting humoral immunity. Meta-analysis was performed on the time to negative urine protein and the time to edema subsidence after treatment. The urine protein negative time and edema subsidence time in the study group were shorter after treatment, but the difference was not notable. This may be related to the lack of contained literature. The dosage of glucocorticoids in the study group was notably lower. This has shown that Huai Qi Huang granule can directly reduce urinary protein, mainly because Chinese wolfberry has the effect of nourishing the liver and kidney, and Rhizoma Polygonatum can nourish the kidney, which is helpful to enhance the renal function of children from the point of view of modern pharmacology. In this study, it was found that the improvement of T lymphoid level and immunoglobulin level in the study group was notably better. It is suggested that combined therapy can better enhance the immune function of children with PNS. It is mainly because Huai Qi Huang granule contains fungus polysaccharides, which can stimulate all aspects of the immune system of children with PNS to help to increase the activity of natural killer cells and T cells, and reduce the activity of B cells. Huai Qi Huang granule can downregulate the inflammatory effect of interleukin-8 and other substances in children's serum, and can also upregulate the anti-inflammatory effect of interleukin-10 [28–30]. At the same time, it has high therapeutic safety and no obvious adverse reactions. It should be recommended as an auxiliary drug for PNS. The conclusion is consistent with the original literature. The result of meta-analysis is not immutable, it is only the result of the comprehensive analysis of the existing data. It is considered that with the continuous inclusion and enrichment of new research data, its conclusions should be updated. In the future, it is necessary to conduct more related randomized controlled trials to verify the efficacy. Therefore, it is recommended to carry out more large-sample, multicenter, high-quality randomized blind studies in strict accordance with the CONSORT statement, to ensure that the follow-up period is long enough, and to provide high-quality research evidence for the secondary evaluation with internationally recognized, objective and transmissible criteria, so as to better evaluate its clinical efficacy and show the value of promotion.

## 5. Conclusion

To sum up, Huai Qi Huang granule associated with hormones has a good clinical effect when treating children with PNS. It can not only enhance the cellular and humoral immune function of children with PNS but also reduce the dosage of prednisone and the occurrence of infection.

## Figures and Tables

**Figure 1:** Illustration of literature screening.

**Figure 2:** Risk of bias chart.

**Figure 3:** Risk of bias summary chart.

**Figure 4:** Forest plot of meta-analysis of infection rate.

**Figure 5:** Forest plot of meta-analysis of recurrence rate.

**Figure 6:** Forest plot of meta-analysis of the incidence of adverse reactions.

**Figure 7:** Forest plot of meta-analysis of serum albumin.

**Figure 8:** Forest plot of meta-analysis of blood cholesterol.

**Figure 9:** Forest plot of meta-analysis of urinary protein negative time.

**Figure 10:** Forest plot of meta-analysis of time for edema to subside.

**Figure 11:** Forest plot of meta-analysis of glucocorticoid dosage.

**Figure 12:** Forest plot of meta-analysis of T lymphocyte level.

**Figure 13:** Forest plot of meta-analysis of immunoglobulin level.

**Figure 14:** Funnel charts of recurrence rate.

**Table 1:** Basic characteristics of literature.

Include the literature	Year of publication	*N* (C/T)	Intervention method		Outcome index	Course of treatment	Stochastic method	Blind or not
			C	T				
Liu and Guo [14]	2020	57/57	Glucocorticoids	Glucocorticoid + Huai Qi Huang granule	①②③④⑤⑦	3 months	The digital parity method	No

Zhiyong and Liu [15]	2016	33/33	Prednisone	Prednisone + Huai Qi Huang granules	①②⑥	3 months	The random number table method	No

Zheng [16]	2015	26/26	Prednisone	Prednisone + Huai Qi Huang granules	③⑦⑧	8 weeks	Not mentioned	No

Yang and Wu [17]	2019	30/30	Glucocorticoids	Glucocorticoid + Huai Qi Huang granule	③④⑧	7 days	A group with odd and even numbers	No

Li et al. [18]	2019	42/43	Prednisone acetate tablets	Prednisone acetate tablets + Huai Qi Huang granules	⑥⑦⑧	3 months	The random number table method	No

Liu et al. [19]	2017	33/35	Prednisone acetate tablets	Prednisone acetate tablets + Huai Qi Huang granules	①②③④⑤⑥⑦	6 months	Not mentioned	No

Geng et al. [20]	2015	23/19	Glucocorticoids	Glucocorticoid + Huai Qi Huang granule	①②③④⑤⑥⑦	3 months	Not mentioned	No

Note: C: control group; T: research group. ① Infection rate; ② Relapse rate; ③ Urinary protein negative time; ④ Edema regression time; ⑤ Glucocorticoid dosage; ⑥ Incidence of adverse reactions; ⑦ T lymphocyte subsets; ⑧ Serum immunoglobulin level.

## Data Availability

The datasets used and analyzed during the current study are available from the corresponding author upon reasonable request.
